# MiR-132 inhibits migration and invasion and increases chemosensitivity of cisplatin-resistant oral squamous cell carcinoma cells via targeting TGF-β1

**DOI:** 10.1080/21655979.2019.1710925

**Published:** 2020-01-07

**Authors:** Liqiang Chen, Qingli Zhu, Lingwei Lu, Yanshan Liu

**Affiliations:** a Department of Oral and Maxillofacial Surgery, The affiliated Hospital of Qingdao University, Qingdao, Shandong, China; b Department of Dental Digital Medicine and 3D Printing Engineering Laboratory, Qingdao University, Qingdao, Shandong, China; c Department of Thyroid Surgery, The affiliated Hospital of Qingdao University, Qingdao, Shandong, China

**Keywords:** Oral squamous cell carcinoma, Chemosensitivity, miR-132, TGF-β1

## Abstract

Numerous findings have demonstrated that MicroRNAs dysregulation plays a key role in many neoplasms, including oral squamous cell carcinoma (OSCC), yet the potential mechanisms of microRNAs in chemo-resistance remain elusive. Here, we analyzed the miR-132 expression in OSCC tissues and OSCC cell lines, and explored it role and mechanisms on invasion and migration and cisplatin (CDDP)-induced cell death. The clinical tissues of 37 patients with OSCCs and paired normal tissues were collected. The miR-132 expression in OSCC tissues and cell lines were detected by reverse transcription-quantitative polymerase chain reation (RT-qPCR). The *in vitro* repopulation models were established to mimic the biological processes of OSCC. The results showed that miR-132 expression was significantly decreased in the OSCC tissues and CDDP resistant OSCC cell line (CAL-27/CDDP). miR-132 mimic inhibited cell proliferation, invasion, migration and enhanced the pro-apoptotic ability of CDDP. On the contrary, downregulation of miR-132 promoted proliferation, invasion, migration and conferred OSCC cell resistance to CDDP-induced apoptosis *in vitro*. The TGF-β1 expression in OSCC tissues and CAL-27/CDDP cells was significantly higher. miR-132 significantly inhibited the TGF-β1/Smad2/3 signals. TGF-β1 upregulation significantly promoted OSCC cell proliferation and resumed OSCC cell chemo-resistance in the miR-132 overexpressing cells, which is contrary to the function of miR-132. In summary, miR-132 acts as a tumor suppressor and exerts a substantial role in inhibiting the proliferation, invasion, and enhanced the chemosensitivity to CDDP of OSCC via regulating TGF-β1/Smad2/3 signals *in vitro*. These observations indicate that miR-132 may be a suitable therapeutic target for the treatment of OSCC.

## Introduction

Head and neck cancer, including oral squamous cell carcinoma (OSCC), is the sixth leading malignancy worldwide, despite significant advances in cancer research over the past few decades [1,2]. Despite a comprehensive treatment concept including surgery, radiation, and chemotherapy, the 5-year survival rate is still only about 50 percent [3,4]. This prognosis has not been improved over the past several years due to the development of distant metastasis, local recurrences and new tumors [5,6]. Consistent with the current guidelines, cisplatin (CDDP)-based chemotherapy remains the gold standard for advanced OSCC and could significantly improve the survival rate [7]. CDDP, which induces apoptotic pathways, was approved by the Food and Drug Administration (FDA) for the treatment of various kinds of solid carcinomas, such as head and neck carcinomas, including OSCC. Although CDDP often leads to therapeutic effects, no substantive progress has been made in overcoming CDDP resistance in a clinical setting due to the numerous resistance mechanisms that cancer cells have [8]. Searching for other mechanisms through which CDDP can exert its apoptotic effects may be the most practical avenue for achieving optimal effectiveness for this drug in a clinical setting.

MiRNAs are a class of small, noncoding RNA molecules, with approximately a length of 19–23 nucleotides [9]. Numerous studies have highlighted the importance of miRNAs in the regulation of gene expression and cellular signaling transduction [10]. In most cases, miRNAs regulate gene expression through direct binding to the matched sites of mRNAs, thus leading to rapid degradation of target mRNAs [11]. It has been firmly established that miRNAs modulate many key cellular functions such as cell proliferation, differentiation, apoptosis, angiogenesis, and stress resistance, and are also involved in a variety of biological processes, such as organism growth, immune regulation and tumorigenesis [10,12]. Recent studies suggested that the acquisition of drug resistance by cancer cells might be modulated via the changes in miRNA levels [13,14]. For instance, miR-27b are downregulated in CDDP resistance OSCC Tca8113 cells, and the overexpression of miR-27b sensitizes Tca8113 cells to CDDP by targeting FZD7 [15]. Upregulation of miR-654-5p promoted proliferation, metastasis, and chemoresistance of OSCC cells through Ras/MAPK signaling [16]. Tian et al. reported that low expression of miR-483-5p were significantly associated with neoadjuvant chemosensitivity and better OSCC patients’ prognosis, and miR-483-5p overexpression reversed the chemoresistance in OSCC cells [17]. LncRNA HOXA11-AS can sensitize human OSCC cells to CDDP by targeting miR-214-3p [18]. Reduced expression of miR-5787 contributes to chemoresistance in TSCC cells by inhibiting the translation of mitochondrial cytochrome oxidase subunit 3 (MT-CO3). The prognostic analysis of TSCC patients showed that the patients with low expression of miR-5787 had poor cisplatin sensitivity and prognosis [19].

miR-132-3p (miR-132) is a known tumor-related miRNA. It is derived from the miR-212/132 cluster and has emerged as key regulator of immune cell development and function [20]. During innate immune activation, miR-132 is induced upon and plays a crucial role in the transcriptional response to pathogenic challenge [21]. however, miR-132 appears to play different roles in various tumor types. miR-132 was reported to be up-regulated and function as a promoter in cancers such as colorectal cancer [22] and pancreatic cancer [23]; while it is down-regulated and functions as a repressor in hepatocellular carcinoma [24], prostate cancer [25], and breast cancer [26]. It has recently found that miR-132 could induce temozolomide resistance and promotes the formation of GIC phenotypes by targeting TUSC3 in glioblastoma initiating cells [27]. MiR-212 could also inhibits CDDP-induced apoptosis by directly targeting AChE-S in NSCLC cells [28]. Mir-132/TGF-β axis is the most extensively studied miRs/TGF-β interaction. It is well established that TGF-β is induced by miR-132 activation in non-small cell lung cancer [29] or inflammation to proliferation during wound healing [30]. However, whether miR-132 is involved in regulating CDDP resistance and invasion in human OSCC cells remains unclear.

In the present study, we aims to investigate the effects and molecular mechanisms of miR-132 on proliferation and invasion of the OSCC cells. In addition, we explored whether human OSCC chemo-resistance can be reversed through targeting miR-132/TGF-β axis.

## Materials and methods

### Sample tissues and cell lines

A total of 37 pairs of OSCC tissues and adjacent normal tissues were collected from Department of Dental Center, the affiliated hospital of Qingdao University. All samples were frozen in liquid nitrogen immediately once dissecting and then were stored at −80°C until further use. Informed consents have been signed by all subjects before clinical surgery. Collection and usage of the samples were reviewed and approved by the affiliated hospital of Qingdao University.

Human OSCC cell lines SCC-9 and CAL-27 were purchased from American Tissue Culture Collection (ATCC; Manassas, VA, USA). Human oral keratinocyte cell line HOK was purchased from BeNa Culture Collection (BNCC; Suzhou, China). Cisplatin [cis-diamminedichloroplatinum (II), CDDP] was purchased from Sigma-Aldrich (Sigma, St. Louis, MO, USA) and dissolved in phosphate-buffered saline (PBS). In accordance with previously described methods, CDDP resistant cell line CAL-27/CDDP was developed from its parental cell line CAL-27 by giving gradually incremental doses of CDDP administration in cell culture medium. All cell lines were cultured in Dulbecco’s Modified Eagle Medium (Life Technologies, Carlsbad, CA, USA) containing 10% fetal bovineserum (FBS; Life Technologies) at 37°C in a humidified with 5% CO_2_ incubator.

### Cell transfection

miRNA mimics or inhibitor targeting miR-132 (miR-132 mimics or miR-132 inhibitor) and their corresponding negative controls (miR-NC or anti-miR-NC) were obtained from RIBOBIO (Guangzhou, China). TGF-β1 overexpressing vector pcDNA3.1-TGF-β1 (TGF-β1) and pcDNA3.1 empty vector (Vector) were synthesized by Genepharma (Shanghai, China). All transfection was performed using Lipofec-tamine 2000 (Invitrogen, Carlsbad, CA, USA). The cells were harvested at 24 h after transfection for the following experiments.

### RNA isolation and qRT-PCR analysis

Trizol reagent (Invitrogen) was used to isolate total RNA from specific tissues and cell lines according to the manufacturer’s protocol. RNA samples were reverse-transcribed into cDNA using a TaqMan MicroRNA Reverse Transcription kit (Applied Biosystems, Foster City, CA, USA) for miR-132 and PrimeScript RT reagent kit (Takara, Dalian, China) for TGF-β1. Then qRT-PCR (Real-Time Quantitative Reverse Transcription PCR) was conducted using TaqMan MicroRNA assays (Applied Biosystems) for miR-132 and SYBR Green Master PCR mix (Applied Biosystems) for TGF-β1 on ABI 7900 system (Applied Biosystems). The expression levels of miR-132 and TGF-β1 were normalized by small RNA U6 (U6) and glyceraldehyde-3-phosphate dehydrogenase (GAPDH), respectively. Expression was calculated using 2^−ΔΔCt^ method. All procedures were performed following the manufacturer’s instructions. The primers used were as follows: GAPDH (Forward, 5ʹ-ATTCCATGGC-ACCGTCAAGGCTGA-3ʹ and Reverse, 5ʹ-TTCTCC-ATGGTGGTGAAGACGCCA-3ʹ); TGF-β1 (Forward, 5ʹ-AGCAAGCTGAAGCTCACCAGT-3ʹ and Reverse, 5ʹ-TTGGCGTAGTACTCTTCGTCG-3ʹ). The primers for miR-132 and U6 were purchased from RiboBio (Guangzhou, China).

### CCK-8 assay

The CDDP resistance and cell proliferation were quantified by CCK-8 assay. For CDDP resistance detection, cells treated with different concentrations of CDDP were planted into 96-well plates (3 × 10^3^). After culture for 48 h, cells were combined with 10 μL reagent of cell counting kit-8 (CCK-8) (Beyotime) for 2 h continuously. Finally, the absorbance value at 450 nm was measured by microplate reader (Bio-Rad, Hercules, CA, USA). Five replicate wells were used for each group. The IC_50_ of CDDP was the CDDP concentration reducing viability by 50%. As for cell proliferation, cells seeded in 96-well plates were cultured for 24 h, 48 h or 72 h, and then examined by CCK-8 as mentioned above.

### Flow cytometry assay

Flow cytometry was carried out for apoptosis analysis by using Fluorescein isothiocyanate (FITC) Annexin V Apoptosis Detection Kits (Invitrogen). In brief, CAL-27 and CAL-27/CDDP cells were incubated for 48 h after transfection. Afterward, cells were trypsinized, washed with PBS, and re-suspended. Next, 5 μL Annexin V-FITC/PI were used to stain apoptotic cells for 15 min in the dark. Subsequently, the apoptotic cells (Annexin V-FITC+ and PI±) were detected using flow cytometer (BD Biosciences, San Jose, CA, USA).

### Transwell assay

Transwells were conducted to detect cell migration and invasion. After 24 h transfection, cells were harvested and re-suspended in serum-free medium. For migration, the cells were placed in the top chamber of a transwell (Corning, NY, USA) and the bottom chamber was filled with DMEM with 10% FBS. After 24 h incubation, the cells migrated to the lower surface of the membrane were fixed with 4% paraformaldehyde (PFA), stained with crystal violet, and photographed using a microscope (Tokyo, Japan) at × 200 magnification. The methods for invasion were similar to the above, except that the upper chamber needed to be coated with Matrigel (Corning) in advance.

### Wound-healing assay

After 24 h transfection, the cells were grown to confluence and scratched with sterile 200 μl pipette tips. Plates were washed twice with PBS to remove detached cells and incubated in the complete growth medium without FBS. Cells migrated into the wounded area, and photographs were taken immediately (0 h) and at 24 h.

### Bioinformatic analysis and luciferase reporter analysis

Online software Targetscan was used to screen putative mRNAs binding to miR-132 and analyze the potential binding sites between miR-132 and 3ʹUTR of TGF-β1. The wild type and mutant sequences of 3ʹUTR of TGF-β1 (TGF-β1-WT and TGF-β1-MUT) containing miR-132 binding sites were inserted into the downstream portion of a dual-luciferase reporter vector. For luciferase assay, 3 × 10^4^ cells were plated and cultured into 24-well plates. CAL-27 cells were co-transfected with miR-132 mimics or miR-NC and TGF-β1-WT or TGF-β1-MUT, respectively. After transfection for 24 h, the luciferase activity was detected using Dual-Luciferase reporter assay system on a luminometer (Promega, Madison, WI, USA).

### Western blot assay

The cells were lysed and proteins were separated using 10% sodium dodecyl sulfate–polyacrylamide gel electrophoresis. After electrophoresis, proteins were electrotransferred onto PVDF membranes (Millipore, Billerica, MA); after the transfer, they were blocked for 2 h in blocking buffer containing 5% nonfat dry milk. Membranes were incubated overnight at 4°C with primary antibodies against TGF-β1, GAPDH, Smad2, Smad3, p-Smad3 and p-Smad2 overnight at 4°C. Then the membranes were washed with TBS with Tween-20 (TBST) for 3 times and were incubated with horseradish peroxidase (HRP)-conjugated secondary antibody. Detection was performed using an ECL chemiluminescence kit (Pierce, Rockford, IL). The film was scanned using ImageQuant software (Molecular Dynamics, Sunnyvale, CA).

### Statistical analysis

All data were shown as mean ± standard deviation (SD). Statistical significance was determined by Student *t* test using the SPSS 17.0 software package. The level of statistical significance was set at p < 0.05.

## Results

### miR-132 expression was significantly decreased in OSCC tissues and OSCC cell lines

The expression of miR-132 was measured in OSCC tissues and paired normal tissues by qRT-PCR. The results showed that miR-132 was significantly down-regulated in OSCC tissues compared with that in normal tissues (Figure 1(a)). In addition, the expression of miR-132 in OSCC cell lines (CAL-27 and SCC-9) was also lower than that of in human oral keratinocytes (HOK) (Figure 1(b)). Moreover, the CDDP-resistant cells (CAL-27/CDDP) expressed much less miR-132 compared to that in CAL-27 cells (Figure 1(b)), suggesting that dysregulation of miR-132 might be associated with CDDP resistance in OSCC cells.

**Figure 1.** Expression of miR-132 in OSCC tissues and cell lines. A. The expression of miR-132 was measured in OSCC tissues and paired normal tissues by qRT-PCR. B. The expression of miR-132 was detected in OSCC cell lines (CAL-27 and SCC-9), human oral keratinocyte cell line (HOK) and CDDP-resistant cell line CAL-27/CDDP. **P < 0.01.

### miR-132 influenced CDDP resistance in OSCC cells

To test the correlation of miR-132 expression and CDDP resistance, miR-132 mimics or miR-NC were transfected into CAL-27 and CAL-27/CDDP cells. First, cell survival rate was measured in CAL-27 and CAL-27/CDDP cells after treatment with different concentrations of CDDP. The result showed that the IC_50_ of CDDP was 1.778 in CAL-27 cells, which was significantly lower than that of in the CAL-27/CDDP cells (5.551) (Figure 2(a)). The qRT-PCR assay showed that the expression of miR-132 was decreased in CAL-27 cells treated with 1 μg/mL CDDP compared the untreated CAL-27 cells (Figure 2(b)). miR-132 was notably upregulated in CAL-27 and CAL-27/CDDP cells transfected with miR-132 mimics compared with miR-NC (Figure 2(c)). And miR-132 upregulation significantly decreased the IC_50_ values of CDDP in both of the CAL-27 and CAL-27/CDDP cells (Figure 2(d,e)). These data implied that miR-132 was able to sensitize OSCC cells to CDDP treatment.

**Figure 2.** Effect of miR-132 overexpression on CDDP resistance in CAL-27 and CAL-27/CDDP cells. (a) The IC_50_ of CDDP in CAL-27 and CAL-27/CDDP cells was analyzed by CCK-8. (b) Expression of miR-132 in CAL-27 cells treated with 1 μg/mL CDDP. (c) The efficiency of miR-132 overexpression was measured in CAL-27 and CAL-27/CDDP cells treated with miR-132 mimics. (d and e) The IC50 of CDDP in CAL-27 and CAL-27/CDDP cells treated with miR-132 mimics was examined using CCK-8. **P < 0.01.

### miR-132 attenuated proliferation, migration and invasion, and promoted apoptosis of OSCC cells

CCK-8 assay showed that overexpression of miR-132 inhibited cell proliferation in CAL-27 and CAL-27/CDDP cells (Figure 3(a,b)). In addition, miR-132 upregulation significantly induced cell apoptosis (Figure 3(c–f)). The number of invaded CAL-27 and CAL-27/CDDP cells transfected with miR-132 mimics was reduced compared with miR-NC transfection by Transwell assay (Figure 3(g)) and Wound-healing assay (Figure 3(h)). Collectively, our findings suggested that miR-132 negatively regulated proliferation, migration, and invasion by functioning as a tumor suppressor in OSCC cells *in vitro*.

**Figure 3.** The role of miR-132 on cell proliferation, apoptosis, migration, and invasion in CAL-27 and CAL-27/CDDP cells. (a and b) CCK-8 was used to measure cell proliferation in CAL-27 and CAL-27/CDDP cells transfected with miR-132 mimics at 24 h, 48 h, and 72 h. (c–f) Flow cytometry was performed to detect cell apoptosis in CAL-27 and CAL-27/CDDP cells transfected with miR-132 mimics. (g) Transwells were used to examine cell migration and invasion in CAL-27 and CAL-27/CDDP cells treated with miR-132 mimics. (h) Quantification of wound gap at 24 h after application of scratch wound are shown. **P < 0.01.

### TGF-β1 was a direct target of miR-132 in OSCC cells

To manifest the underlying mechanisms of miR-132 expression on cell growth and invasion in OSCC cells, we screened the putative targets of miR-132 using bioinformatics tool Targetscan. The binding sites of miR-132 and 3ʹUTR of TGF-β1 are displayed in Figure 4(a). The sequences containing the WT or MUT 3ʹUTR of TGF-β1 (TGF-β1-WT and TGF-β1-MUT) (Figure 4(a)) were inserted into luciferase reporter plasmid, and the fusion plasmid together with miR-132 mimics or miR-NC were cotransfected in CAL-27 cells. As shown in Figure 4(b), when CAL-27 cells were transfected with the TGF-β1-WT 3ʹUTR, co-transfection of miR-132 mimics significantly inhibited luciferase activity. In contrast, the influence of miR-132 mimics was not obvious in CAL-27 cells co-transfected with TGF-β1-MUT 3ʹUTR. Also, the TGF-β1 mRNA expression was greatly strengthened in CAL-27 and CAL-27/CDDP cells compared with that in HOK cells (Figure 4(c)). After treatment with 1 μg/mL CDDP, the relative TGF-β1 mRNA (Figure 4(d)) and TGF-β1 protein expression (Figure 4(e)) were rapidly enhanced in CAL-27 cells compared with those in untreated cells.

**Figure 4.** Relationship between miR-132 and TGF-β1 in CAL-27 cells. (a) Putative binding sites of TUG1 and miR-132 are shown. (b) Luciferase activity was detected in CAL27 cells co-transfected with TGF-β1 WT or TGFβ1 MUT and miR-132 or miR-NC. (c) The miR-132 mRNA expression was measured in HOK, CAL-27, and CAL-27/CDDP cells. (d and e) The TGF-β1 mRNA expression and TGF-β1 protein expression were measured in CAL-27 cells treated with 1 μg/mL CDDP. (f) The enrichment of TGF-β1 was investigated in CAL27 cells transfected with miR-132 mimics or miR-132 inhibitor. (g) The expression of SMAD family proteins was examined in CAL27 cells transfected with miR-132 mimics or miR-132 inhibitor by western blot assay. (h) The level of TGF-β1 was detected in OSCC tissues and paired normal tissues. (i) The correlation of TGF-β1 expression and miR-132 expression was analyzed. *P < 0.05, **P < 0.01.

Next, we investigated the effects of miR-132 on TGF-β1 mRNA expression in CAL-27 cells. The data indicated that the TGF-β1 mRNA expression increased sharply in the miR-132 inhibitor groups compared to the anti-miR-NC groups. However, TGF-β1 mRNA expression was very weak in the miR-132 mimics groups compared with that in the miR-NC groups (Figure 4(f)). Moreover, the TGF-β1 signal related proteins p-Smad2 and p-Smad3 were also significantly upregulated in the miR-132 inhibitor groups compared with that in the anti-miR-NC groups. The p-Smad2 and p-Smad3 protein were also makedly decreased in CAL-27 cells transfected with miR-132 mimics compared with miR-NC (Figure 4(g)). Additionally, the forced expression of TGF-β1 in OSCC tissues was negatively correlated with the expression of miR-132 (Figure 4(h,i)). The above data suggest that miR-132 regulated the expression of TGF-β1 at the transcriptional and translational levels by directly binding to putative TGF-β1 3ʹUTR regions.

### miR-132 enhances CDDP chemosensitivity by targeting TGF-β1 in OSCC cells

To verify the interaction of miR-132 and TGF-β1 on CDDP resistance, CAL-27 and CAL-27/CDDP cells were transfected with miR-132 mimics, miR-NC and miR-132 mimics + TGF-β1. The transfection efficacy was validated at the transcriptional level and protein level. As exhibited in Figure 5(a–c), the mRNA expression and protein expression of TGF-β1 were decreased in CAL-27 and CAL-27/CDDP cell lines transfected with miR-132 mimics compared to miR-NC. On the contrary, the TGF-β1 mRNA and TGF-β1 protein expression were recovered in the two cell lines transfected with miR-132 mimics + TGF-β1. In addition, gain-of-function experiments showed that upregulation of miR-132 impeded CDDP resistance, measured by the IC50 to CDDP. Nevertheless, upregulation of miR-132 reversed the suppressive role of miR-132 overexpression in both CAL-27 and CAL-27/CDDP cells (Figure 5(d,e)). These data suggested that miR-132 regulated CDDP chemosensitivity by binding to TGF-β1 directly in CAL-27 and CAL-27/CDDP cells.

**Figure 5.** Effect of TGF-β1 overexpression on miR-132-mediated CDDP resistance in CAL-27 and CAL-27/CDDP cells. (a-c) TGFβ1 expression was measured in the miR-132 overexpressing CAL-27 and CAL-27/CDDP cells treated with pcDNA-TGFβ1 at the mRNA level (a) and protein level (b and c). (d and e) The IC_50_ of CDDP in the CAL-27 and CAL-27/CDDP cells treated with miR-132 mimics + TGFβ1, miR-132 mimics + vector, miR-132 mimics, or miR-NC was examined by CCK-8. **P < 0.01.

### miR-132 regulates cell proliferation, apoptosis, migration, and invasion in OSCC cells by targeting TGF-β1

To further define the mechanism of miR-132 function in CAL-27 and CAL-27/CDDP cells, cell proliferation, apoptosis, migration, and invasion were detected in CAL-27 and CAL-27/CDDP cell lines. As shown in Figure 6(a,b), co-transfection of miR-132 mimics and TGF-β1 restored the inhibited role of miR-132 mimic transfection in CAL-27 and CAL-27/CDDP cells. Furthermore, miR-132 mimics rapidly induced cell apoptosis in both of the cells, while miR-132 mimics + TGF-β1 transfection reduced the amount of apoptotic cells (Figure 6(c)). As for cell migration and invasion, miR-132 mimics + TGF-β1 transfection the reversed the migrative and invasive ability of the miR-132 expressing cells (Figure 6(d,e)).

**Figure 6.** Effect of TGF-β1 overexpression on miR-132-regulated cell proliferation, apoptosis, migration and invasion. CAL-27 and CAL-27/CDDP cells were transfected with miR-132 mimics + TGF-β1, miR-132 mimics + vector, miR-132 mimics, or miR-NC for 24 h. (a,b) Cell proliferation, (c) apoptosis, (d) cell invasion and (e) cell migration were measured by CCK-8, flow cytometry, transwell, or wound healing assay, respectively. *P < 0.05, **P < 0.01.

## Discussion

The prognosis of OSCC is poor due to the complex metastasis mechanism and chemical resistance. Thus, an understanding of the tumor growth, metastasis, and drug resistance mechanisms is indispensable, and a systemic attempt is necessary to improve the outcome of OSCC patients. In the present study, we determined that miR-132 acted as a tumor suppressor and sensitized cells to CDDP in OSCC. Also, the target TGF-β1 of miR-132 was confirmed here, which revealed a novel biological axis of miR-132/TGF-β1 in CDDP chemosensitivity and cell proliferation, migration, and invasion in OSCC cells.

It was well-demonstrated that ectopic expression of miR-132 played a crucial role on tumor development and metastasis in human cancers. For example, miR-132 level was obviously lower in human bladder cancer and overexpression of miR-132 inhibited cell proliferation and invasion to some extent [31]. miR-132 overexpression notably reduced cell proliferation and colony formation, and promoted cell apoptosis in breast cancer cells [32]. In our study, miR-132 was down-regulated in OSCC tissues and OSCC cells, miR-132 overexpression inhibited cell proliferation, migration, and invasion, and accelerated apoptosis in OSCC, suggesting that miR-132 is the tumor suppressor.

Cheng et al. reported that miR-132 induced temozolomide resistance and promotes the formation of cancer stem cell phenotypes by targeting TUSC3 in glioblastoma [27]. In gastric cancer, the enhanced miR-132 expression correlated chemo-resistance in GC patients, and miR-132 promoted CDDP resistance in Lgr5^+^ GCSCs in vitro and in vivo [33]. However, miR-132 overexpression increase the sensitivity of SKOV3/CDDP cells to CDDP, and inhibit cell invasion and metastasis [34]. In our study, CDDP-resistant OSCC cell lines showed lower miR-132 expression, enforced miR-132 expression in the CDDP-resistant OSCC cells restored the sensitivity of DDP resistant cells to CDDP.

Transforming growth factor β (TGF-β) is a 25 kDa disulfide-linked dimeric protein that has 3 isoforms: TGF-β1, -β2, and -β3. TGF-β is a secreted cytokine that regulates cell proliferation, migration, and the differentiation of a plethora of different cell types [35]. Consistent with these findings, TGF-β plays a key role in controlling embryogenic development, inflammation, and tissue repair, as well as in maintaining adult tissue homeostasis [36,37]. TGF-β overexpression has been demonstrated in both animal and human tumor models and is seen clinically in many tumors including cancers of the breast, colon, esophagus, stomach, liver, lung, kidney, pancreas, prostate, brain, and malignant melanoma, as well as certain hematological malignancies [38]. Studies *in vivo* and *in vitro* showed that TGF-β1 overexpression resulted in increased cell proliferation and invasiveness, and enhanced metastatic potential [39–42]. In addition, silence of TGF-β1 enhanced the sensitivity to CDDP of A549/CDDP through inducing the reversal of EMT and inhibiting the expression of resistance-associated proteins [43]. Takayama et al. reported that inhibition of TGF-β1 suppresses motility and invasiveness of OSCC cells via modulation of integrins and matrix-metalloproteinases in OSCC cells [44].

Function assays showed that miR-132 overexpression in TPC1 cells inhibited cell proliferation, migration, and invasion through targeting FOXA1 [45]. In ovarian cancer cells, miR-132 suppresses the cell proliferation, invasion, migration by targeting E2F5 [46]. Introduction of miR-132 significantly suppressed the migration and invasion of lung cancer cells *in vitro* by targeting SOX4 [47]. Wei et al. reported that miR-132 may played a suppressive role in the metastasis of BC cells via TGFβ1/Smad2 signaling pathway [31]. Overexpression of miR-132/212 inhibited TGF-β-induced EMT in Vcap and Lncap cells at both the mRNA and protein expression levels [48]. In addition, miR-212/132 functions as tumor suppressor by targeting Smad2 in cervical cancer [49]. In the present study, we showed that the expression level of TGF-β1 was significantly increased in OSCC tissues and its expression was inversely correlated with miR-132 expression in clinical OSCC tissues. Of note, we found that upregulation of TGF-β1 have reversed the effect of miR-132 overexpression on the OSCC cell lines. These results suggested that miR-132 exerted tumor suppressor role in OSCC by targeting TGF-β1. Moreover, we found that miR-132 overexpression inhibited TGF-β1 protein expression, and vice versa, and downregulation of miR-132 conferred chemoresistance to OSCC cells by TGF-β1 overexpression.

## Conclusion

We demonstrated that miR-132 inhibited cell proliferation and invasion, and augmented the chemosensitivity to CDDP in OSCC cells *in vitro* by targeting TGF-β1/Smad2/3 signal. Our findings suggested that the miR-132/TGF-β1 axis might be a promising prognostic and therapeutic target in OSCC.

## Article highlights

- miR-132 expression is decreased in OSCC tissues and CDDP resistant OSCC cell line.
- miR-132 negatively regulated TGF-β1/Smad2/3 signals in OSCC cells.
- miR-132 inhibited proliferation and invasion, and enhanced the chemosensitivity in OSCC cells
- miR-132 enhanced the chemosensitivity to CDDP via targeting TGF-β1/Smad2/3 signals in OSCC cells.

## References

[1] Choi S, Myers J. Molecular pathogenesis of oral squamous cell carcinoma: implications for therapy. J Dent Res. 2008;87:14.1809688910.1177/154405910808700104

[2] Rivera C, Venegas B. Histological and molecular aspects of oral squamous cell carcinoma (Review). Oncol Lett. 2014;8:7–11.2495921110.3892/ol.2014.2103PMC4063640

[3] Parkin DM, Bray F, Ferlay J, et al. Global cancer statistics, 2002. CA Cancer J Clin. 2005;55:74–108.1576107810.3322/canjclin.55.2.74

[4] Gedlicka C, Formanek M, Selzer E, et al. Phase II study with docetaxel and cisplatin in the treatment of recurrent and/or metastatic squamous cell carcinoma of the head and neck. Oncology. 2002;63:145–150.1223944910.1159/000063809

[5] Bettendorf O, Piffko J, Bankfalvi A. Prognostic and predictive factors in oral squamous cell cancer: important tools for planning individual therapy? Oral Oncol. 2004;40:110–119.1469323310.1016/j.oraloncology.2003.08.010

[6] Rogers SN, Brown JS, Woolgar JA, et al. Survival following primary surgery for oral cancer. Oral Oncol. 2009;45:201–211.1867495910.1016/j.oraloncology.2008.05.008

[7] Gibson MK, Li Y, Murphy B, et al.; Eastern Cooperative Oncology Group. Randomized phase III evaluation of cisplatin plus fluorouracil versus cisplatin plus paclitaxel in advanced head and neck cancer (E1395): an intergroup trial of the Eastern Cooperative Oncology Group. J Clin Oncol. 2005;23:3562–3567.1590866710.1200/JCO.2005.01.057

[8] Galluzzi L, Senovilla L, Vitale I, et al. Molecular mechanisms of cisplatin resistance. Oncogene. 2012;31:1869–1883.2189220410.1038/onc.2011.384

[9] Esquela-Kerscher A, Slack FJ. Oncomirs - microRNAs with a role in cancer. Nat Rev Cancer. 2006;6:259–269.1655727910.1038/nrc1840

[10] Baltimore D, Boldin MP, O’Connell RM, et al. MicroRNAs: new regulators of immune cell development and function. Nat Immunol. 2008;9:839–845.1864559210.1038/ni.f.209

[11] Pereira DM, Rodrigues PM, Borralho PM, et al. Delivering the promise of miRNA cancer therapeutics. Drug Discov Today. 2013;18:282–289.2306409710.1016/j.drudis.2012.10.002

[12] Plasterk RH. Micro RNAs in animal development. Cell. 2006;124:877–881.1653003210.1016/j.cell.2006.02.030

[13] Liu T, Zhang X, Du L, et al. Exosome-transmitted miR-128-3p increase chemosensitivity of oxaliplatin-resistant colorectal cancer. Mol Cancer. 2019;18:43.3089016810.1186/s12943-019-0981-7PMC6423768

[14] Rezaei Z, Sebzari A, Kordi-Tamandani DM, et al. Involvement of the dysregulation of miR-23b-3p, miR-195-5p, miR-656-5p, and miR-340-5p in trastuzumab resistance of HER2-positive breast cancer cells and system biology approach to predict their targets involved in resistance. DNA Cell Biol. 2019;38:184–192.3070233710.1089/dna.2018.4427

[15] Liu B, Cao G, Dong Z, et al. Effect of microRNA-27b on cisplatin chemotherapy sensitivity of oral squamous cell carcinoma via FZD7 signaling pathway. Oncol Lett. 2019;18:667–673.3128954010.3892/ol.2019.10347PMC6540118

[16] Lu M, Wang C, Chen W, et al. miR-654-5p targets GRAP to promote proliferation, metastasis, and chemoresistance of oral squamous cell carcinoma through Ras/MAPK signaling. DNA Cell Biol. 2018;37:381–388.2936470510.1089/dna.2017.4095

[17] Tian T, Lv X, Pan G, et al. Long noncoding RNA MPRL promotes mitochondrial fission and cisplatin chemosensitivity via disruption of pre-miRNA processing. Clin Cancer Res. 2019;25:3673–3688.3088593910.1158/1078-0432.CCR-18-2739PMC8725174

[18] Wang X, Li H, Shi J. LncRNA HOXA11-AS promotes proliferation and cisplatin resistance of oral squamous cell carcinoma by suppression of miR-214-3p expression. Biomed Res Int. 2019;2019:8645153.3127598810.1155/2019/8645153PMC6558628

[19] Chen W, Wang P, Lu Y, et al. Decreased expression of mitochondrial miR-5787 contributes to chemoresistance by reprogramming glucose metabolism and inhibiting MT-CO3 translation. Theranostics. 2019;9:5739–5754.3153451610.7150/thno.37556PMC6735381

[20] Wanet A, Tacheny A, Arnould T, et al. miR-212/132 expression and functions: within and beyond the neuronal compartment. Nucleic Acids Res. 2012;40:4742–4753.2236275210.1093/nar/gks151PMC3367188

[21] Lagos D, Pollara G, Henderson S, et al. miR-132 regulates antiviral innate immunity through suppression of the p300 transcriptional co-activator. Nat Cell Biol. 2010;12:513–519.2041886910.1038/ncb2054

[22] Zhang M, Li Y, Wang H, et al. LncRNA SNHG5 affects cell proliferation, metastasis and migration of colorectal cancer through regulating miR-132-3p/CREB5. Cancer Biol Ther. 2019;20:524–536.3039576710.1080/15384047.2018.1537579PMC6422517

[23] Park JK, Henry JC, Jiang J, et al. miR-132 and miR-212 are increased in pancreatic cancer and target the retinoblastoma tumor suppressor. Biochem Biophys Res Commun. 2011;406:518–523.2132966410.1016/j.bbrc.2011.02.065PMC3069485

[24] Zhang X, Tang W, Li R, et al. Downregulation of microRNA-132 indicates progression in hepatocellular carcinoma. Exp Ther Med. 2016;12:2095–2101.2769869810.3892/etm.2016.3613PMC5038555

[25] Formosa A, Lena AM, Markert EK, et al. DNA methylation silences miR-132 in prostate cancer. Oncogene. 2013;32:127–134.2231029110.1038/onc.2012.14

[26] Zhang ZG, Chen WX, Wu YH, et al. MiR-132 prohibits proliferation, invasion, migration, and metastasis in breast cancer by targeting HN1. Biochem Biophys Res Commun. 2014;454:109–114.2545036510.1016/j.bbrc.2014.10.049

[27] Cheng ZX, Yin WB, Wang ZY. MicroRNA-132 induces temozolomide resistance and promotes theformation of cancer stem cell phenotypes by targeting tumor suppressorcandidate 3 in glioblastoma. Int J Mol Med. 2017;40:1307–1314.2890139010.3892/ijmm.2017.3124PMC5627876

[28] Lu L, Xuejin Z, Bo Z, et al. Synaptic acetylcholinesterase targeted by microRNA-212 functions asa tumor suppressor in non-small cell lung cancer. Int J Biochem Cell Biol. 2013;45:2530–2540.2397400810.1016/j.biocel.2013.08.007

[29] Zhang JX, Zhai JF, Yang XT, et al. MicroRNA-132 inhibits migration, invasion and epithelial-mesenchymal transition by regulating TGFβ1/Smad2 in human non-small cell lung cancer. Eur Rev Med Pharmacol Sci. 2016;20:3793–3801.27735039

[30] Li D, Wang A, Liu X, et al. MicroRNA-132 enhances transition from inflammation to proliferation during wound healing. J Clin Invest. 2015;125:3008–3026.2612174710.1172/JCI79052PMC4563743

[31] Wei XC, Lv ZH. MicroRNA-132 inhibits migration, invasion and epithelial-mesenchymal transition via TGFβ1/Smad2 signaling pathway in human bladder cancer. Onco Targets Ther. 2019;12:5937–5945.3141359110.2147/OTT.S201731PMC6662166

[32] Xie M, Fu Z, Cao J, et al. MicroRNA-132 and microRNA-212 mediate doxorubicin resistance by down-regulating the PTEN-AKT/NF-κB signaling pathway in breast cancer. Biomed Pharmacother. 2018;102:286–294.2956754210.1016/j.biopha.2018.03.088

[33] Zhang L, Guo X, Zhang D, et al. Upregulated miR-132 in Lgr5_+_ gastric cancer stem cell-like cells contributes to cisplatin-resistance via SIRT1/CREB/ABCG2 signaling pathway. Mol Carcinog. 2017;56:2022–2034.2838376310.1002/mc.22656

[34] Zhang XL, Sun BL, Tian SX, et al. MicroRNA-132 reverses cisplatin resistance and metastasis in ovarian cancer by the targeted regulation on Bmi-1. Eur Rev Med Pharmacol Sci. 2019;23:3635–3644.3111498810.26355/eurrev_201905_17787

[35] Zhang Y, Alexander PB, Wang XF. TGF-β family signaling in the control of cell proliferation and survival. Cold Spring Harb Perspect Biol. 2017;3:9.10.1101/cshperspect.a022145PMC537805427920038

[36] Pastushenko I, Brisebarre A, Sifrim A, et al. Identification of the tumour transition states occurring during EMT. Nature. 2018;556:463–468.2967028110.1038/s41586-018-0040-3

[37] Wiener Z, Band AM, Kallio P, et al. Oncogenic mutations in intestinal adenomas regulate bim-mediated apoptosis induced by TGF-β. Proc Natl Acad Sci U S A. 2014;111:E2229–2236.2482588910.1073/pnas.1406444111PMC4040601

[38] Fabregat I, Fernando J, Mainez J, et al. TGF-beta Signaling in Cancer Treatment. Curr Pharm Des. 2014;20:2934–2947.2394436610.2174/13816128113199990591

[39] Moon H, Ju HL, Chung SI, et al. Transforming growth factor-β promotes liver tumorigenesis in mice via up-regulation of snail. Gastroenterology. 2017;153:1378–1391.2873483310.1053/j.gastro.2017.07.014

[40] Gencer S, Oleinik N, Kim J, et al. TGF-β receptor I/II trafficking and signaling at primary cilia are inhibited by ceramide to attenuate cell migration and tumor metastasis. Sci Signal. 2017;10:eaam7464.10.1126/scisignal.aam7464PMC581898929066540

[41] Luo Y, Huang K, Zheng J, et al. TGF-β1 promotes cell migration in hepatocellular carcinoma by suppressing reelin expression. Gene. 2019;688:19–25.3044734510.1016/j.gene.2018.11.033

[42] Cui W, Meng W, Zhao L, et al. TGF-β-induced long non-coding RNA MIR155HG promotes the progression and EMT of laryngeal squamous cell carcinoma by regulating the miR-155-5p/SOX10 axis. Int J Oncol. 2019;54:2005–2018.3108104310.3892/ijo.2019.4784PMC6521927

[43] Wang J, Chen Y, Xiang F, et al. Suppression of TGF-β1 enhances chemosensitivity of cisplatin-resistant lung cancer cells through the inhibition of drug-resistant proteins. Artif Cells Nanomed Biotechnol. 2018;46:1505–1512.2891867310.1080/21691401.2017.1374285

[44] Takayama S, Hatori M, Kurihara Y, et al. Inhibition of TGF-beta1 suppresses motility and invasiveness of oral squamous cell carcinoma cell lines via modulation of integrins and down-regulation of matrix-metalloproteinases. Oncol Rep. 2009;21:205–210.19082463

[45] Chen X, Li M, Zhou H, et al. miR-132 targets FOXA1 and exerts tumor-suppressing functions in thyroid cancer. Oncol Res. 2019;27:431–437.2952322110.3727/096504018X15201058168730PMC7848280

[46] Tian H, Hou L, Xiong YM, et al. miR-132 targeting E2F5 suppresses cell proliferation, invasion, migration in ovarian cancer cells. Am J Transl Res. 2016;8:1492–1501.27186275PMC4859634

[47] Li Y, Zu L, Wang Y, et al. miR-132 inhibits lung cancer cell migration and invasion by targeting SOX4. J Thorac Dis. 2015;7:1563–1569.2654360310.3978/j.issn.2072-1439.2015.09.06PMC4598519

[48] Fu W, Tao T, Qi M, et al. MicroRNA-132/212 upregulation inhibits TGF-β-mediated epithelial-mesenchymal transition of prostate cancer cells by targeting SOX4. Prostate. 2016;76:1560–1570.2752711710.1002/pros.23241

[49] Zhao JL, Zhang L, Guo X, et al. miR-212/132 downregulates SMAD2 expression to suppress the G1/S phase transition of the cell cycle and the epithelial to mesenchymal transition in cervical cancer cells. IUBMB Life. 2015;67:380–394.2598833510.1002/iub.1381

